The article "MicroRNA-30d promotes angiogenesis and tumor growth via MYPT1/c-JUN/VEGFA pathway and predicts aggressive outcome in prostate cancer" was retracted in 2023. Reasons: duplicated images; unreliable results or conclusions.

# MicroRNA-30d promotes angiogenesis and tumor growth via MYPT1/c-JUN/VEGFA pathway and predicts aggressive outcome in prostate cancer

**DOI:** 10.1186/s12943-017-0615-x

**Published:** 2017-02-27

**Authors:** Zhuo-yuan Lin, Guo Chen, Yan-qiong Zhang, Hui-chan He, Yu-xiang Liang, Jian-heng Ye, Ying-ke Liang, Ru-jun Mo, Jian-ming Lu, Yang-jia Zhuo, Yu Zheng, Fu-neng Jiang, Zhao-dong Han, Shu-lin Wu, Wei-de Zhong, Chin-Lee Wu

**Affiliations:** 1 Department of Urology, Guangdong Key Laboratory of Clinical Molecular Medicine and Diagnostics, Guangzhou First People’s Hospital, Guangzhou Medical University, Guangzhou, 510180 China; 2 Department of Urology, The Second Affiliated Hospital of Guangzhou Medical University, Guangzhou Medical University, Guangzhou, 510260 China; 3 Institute of Chinese Materia Medica, China Academy of Chinese Medical Sciences, Beijing, 100700 China; 4 Guangdong Provincial Institute of Nephrology, Nanfang Hospital, Southern Medical University, Guangzhou, 510515 China; 5 Urology Key Laboratory of Guangdong Province, The First Affiliated Hospital of Guangzhou Medical University, Guangzhou Medical University, Guangzhou, 510230 China; 6 Graduate school of Jinan University, Guangzhou, 510632 China; 7 Department of Pathology, Massachusetts General Hospital and Harvard Medical School, Boston, MA 02114 USA; 8 Department of Urology, Massachusetts General Hospital and Harvard Medical School, Boston, MA 02114 USA

**Keywords:** Prostate cancer, MicroRNA-30d, Myosin phosphatase targeting subunit 1, Prognosis, Tumor angiogenesis

## Abstract

**Background:**

Even though aberrant expression of microRNA (miR)-30d has been reported in prostate cancer (PCa), its associations with cancer progression remain contradictory. The aim of this study was to investigate clinical significance, biological functions and underlying mechanisms of miR-30d deregulation in PCa.

**Methods:**

Involvement of miR-30d deregulation in malignant phenotypes of PCa was demonstrated by clinical sample evaluation, and in vitro and in vivo experiments. The mechanisms underlying its regulatory effect on tumor angiogenesis were determined.

**Results:**

miR-30d over-expression was observed in both PCa cells and clinical specimens. High-miR-30d was distinctly associated with high pre-operative PSA and Gleason score, advanced clinical and pathological stages, positive metastasis and biochemical recurrence (BCR), and reduced overall survival of PCa patients. Through gain- and loss-of-function experiments, we found that miR-30d promoted PCa cell proliferation, migration, invasion, and capillary tube formation of endothelial cells, as well as in vivo tumor growth and angiogenesis in a mouse model. Simulation of myosin phosphatase targeting subunit 1 (MYPT1), acting as a direct target of miR-30d, antagonized the effects induced by miR-30d up-regulation in PCa cells. Notably, miR-30d/MYPT1 combination was identified as an independent factor to predict BCR of PCa patients. Furthermore, miR-30d exerted its pro-angiogenesis function, at least in part, by inhibiting MYPT1, which in turn, increased phosphorylation levels of c-JUN and activated VEGFA-induced signaling cascade in endothelial cells.

The article "MicroRNA-30d promotes angiogenesis and tumor growth via MYPT1/c-JUN/VEGFA pathway and predicts aggressive outcome in prostate cancer" was retracted in 2023. Reasons: duplicated images; unreliable results or conclusions.

**Conclusions:**

miR-30d and/or its target gene MYPT1 may serve as novel prognostic markers of PCa. miR-30d promotes tumor angiogenesis of PCa through MYPT1/c-JUN/VEGFA pathway.

**Electronic supplementary material:**

The online version of this article (doi:10.1186/s12943-017-0615-x) contains supplementary material, which is available to authorized users.

## Background

As a unique and heterogeneous disease, prostate cancer (PCa) represents the second most frequent malignancy in men and a major cause of cancer-related deaths worldwide [1]. The incidence and mortality of PCa are both rising steadily in multiple countries. For example, approximately 220,000 American men were diagnosed as PCa and 27,000 died of this cancer in 2015 [2]. Although serum prostate-specific antigen (PSA) has been extensively used as a diagnostic biomarker for clinical screening of patients with PCa, the specificity of this parameter is relative low (about 25 ~ 40%) when it is between 4.0–10.0 ng/mL, leading to a high rate of negative biopsy and overtreatment [3]. To overcome this defect, accumulating studies have developed multiple risk stratification systems, which integrate several available clinical and pathological parameters (such as PSA levels, Gleason score, and clinical and pathological stages) [4]. Unfortunately, the efficiencies of these systems on early diagnosis and outcome prediction are still unsatisfactory. Therefore, there is an urgent clinical need to explore molecular mechanisms underlying tumor development and progression of PCa, in order to identify novel biomarkers which can distinguish indolent disease from aggressive disease, and to provide potential therapeutic targets for the improvement of patients’ outcome.

MicroRNAs (miRNAs), a class of highly conserved, small non-coding RNA molecules with 18–25 nucleotides in length, function as post-transcriptional regulators of gene expression via directly degrading mRNA or indirectly repressing protein translation [5]. Growing evidence show that miRNA deregulation is implicated into multiple human cancers through regulating a wide range of pathological processes [6]. Functionally, miRNAs act as either oncogenes or as tumor suppressors due to the different cellular contexts of malignancies [7]. miR-30d, together with miR-30a, b, c and e, belongs to the human miR-30 family and is localized to chromosomal region 8q24 [8]. Accumulating studies have revealed that miR-30d plays a crucial role in various physiological processes in normal and malignant tissues, including cell development, proliferation, apoptosis, migration, invasion and angiogenesis [9, 10].

The article "MicroRNA-30d promotes angiogenesis and tumor growth via MYPT1/c-JUN/VEGFA pathway and predicts aggressive outcome in prostate cancer" was retracted in 2023. Reasons: duplicated images; unreliable results or conclusions.

There are still controversies about the roles of miR-30d in human PCa. A previous study of Kobayashi et al. [11] showed that miR-30d might serve as a potential unfavorable prognostic factor in PCa; Liang et al. [12] indicated that miR-30d expression was up-regulated in high Gleason score (≥8) PCa; In contrast, Xuan et al. [13] reported that it exhibited tumor suppressive properties in this cancer; Xu et al. [14] observed the downregulation of miR-30d in PCa; Kumar et al. [15] indicated that miR-30d levels in metastatic castration resistant PCa (CRPC) were significantly reduced when compared to healthy prostate tissues, and were inversely correlated with AR activity. These different findings might be caused by patients’ heterogenicity and various experimental platforms. To determine the exact role of miR-30d in PCa, we here examined the expression patterns of miR-30d in PCa cell lines and clinical tissue samples, and then verified its clinical relevance and functions on various malignant phenotypes of PCa cells using both gain- and loss-of-function analyses. Moreover, we identified direct target genes of this miRNA and further investigated the molecular mechanisms underlying the pro-angiogenesis of miR-30d in PCa. (Additional file 1: Figure S1).

## Methods

### Ethic statement

This study was approved by the human study ethics (IRB) committees at MGH, Boston, MA and the Ministry of Public Health of P. R. China. All specimens were handled and made anonymous according to the ethical and legal standards.

All animal experiments in this study were performed in compliance with the guidelines of the Institute for Laboratory Animal Research at Guangzhou Medical University, Guangzhou, P. R. China.

### Patients and tissue samples

This study used the same cohorts of patients and tissue samples with our previous study [16]. Detailed information is provided in Additional file 2: File S1-section 1.

### Cell culture

Normal human prostate epithelial cells (PREC) and two human PCa cell lines LNCaP and DU145 were used in this study. Detailed information is provided in Additional file 2: File S1-section 2.

### Animals

Twenty BALB/c nude mice (4 ~ 5-week-old males) were purchased from Guangdong Medical Laboratory Animal Center and were housed five per cage in wire-top cages with sawdust bedding in an isolated, clean, air-conditioned room at a temperature of 25–26 °C and a relative humidity of ~50%, lit 12 h/day.

The article "MicroRNA-30d promotes angiogenesis and tumor growth via MYPT1/c-JUN/VEGFA pathway and predicts aggressive outcome in prostate cancer" was retracted in 2023. Reasons: duplicated images; unreliable results or conclusions.

### Cell transfection

To enforce and inhibit the expression of miR-30d in PCa cells, the miR-30d precursor and sh-miR-30d construct were respectively transfected according to the protocol described previously [16–18]. For the miR-30d precursor (miR-30d), the coding sequence of miR-30d was cloned into the pMIRNA1 lentivectors (Human pre-microRNA Expression Construct Lenti-miR-30d MI0000255, Cat No: PMIRH30dPA-1, SBI, USA; The coding sequence of miR-30d is provided in Additional file 2: File S1-section 3); For negative control precursor (miR-NC), pCDH-CMV-Scramble hairpin-EF1-copGFP (CD511B-1) was purchased from the same vendor (Cat No: PMIRH000PA-1, SBI, USA); For sh-miR-30d (sh-30d) and anti-control (sh-NC) constructs, the miRZip-30d sh-miR-30d microRNA construct (Cat No: MZIP30d-PA-1) and miRZip control vectors (Cat No: MZIP000-PA-1) were designed and cloned by SBI, USA. To package these constructs, 293TN cells were transfected with miR-30d/miR-NC or sh-30d/sh-NC by pPACKH1 Packaging Plasmid Mix (Cat No: LV500A-1, SBI, USA), and then after three days, the virus particles were collected according to the packaging protocol of SBI with the Lenti-Concentin Virus Precipitation Solution (Cat No: LV810A-1, SBI, USA). DU145 and LNCaP cells were infected with TransDux virus transduction reagent (Cat No: LV850A-1, SBI, USA). The infected cells were isolated with a flow cytometer and cultured in 96-well plates.

The myosin phosphatase targeting protein 1 (MYPT1) coding sequence cloned into pLL3.7-CMV-IRES-puro-Vector (Provided by Huijun company of China)/blank vector (NC), and shRNA-targeting human MYPT1 (sh-MYPT1, Cat. No: GV248, Genechem, China) and the shRNA non-targeting (sh-NC, Cat. No: CON077, Genechem, China) were transfected into PCa cells using Lipofectamine 2000 Reagent (Cat. No: 11668019, Invitrogen, USA) according to the manufacturer’s protocol. Forty-eight hours after the transfection, PCa cells were collected and used for the functional analyses.

### Cell viability assay

Cell viabilities were detected by CCK-8 assay according to the protocol of our previous studies [16–18].

### Cell invasion and migration assays

Cell invasion and migration were respectively detected by the Transwell and the scratch wound-healing motility assay according to the protocol of our previous studies [16–18].

### Tube formation

HUVECs (2 × 10^4^) were plated onto matrigel-coated (10 mg/ml, BD Pharmingen, San Jose, CA) 12-well plates with condition media of LNCaP and DU145 cells. After 12 hours of the incubation at 37 °C, HUVECs were fixed with 4% paraformaldehyde and the formation of capillary-like structures was captured under a light microscope (OLYMPUS CKX41, U-CTR30-2, Japan). The number of branch points of the tube structures, as the degree of angiogenesis, was counted in three fields at 100× magnification.

The article "MicroRNA-30d promotes angiogenesis and tumor growth via MYPT1/c-JUN/VEGFA pathway and predicts aggressive outcome in prostate cancer" was retracted in 2023. Reasons: duplicated images; unreliable results or conclusions.

### In vivo tumor angiogenesis assay

For the in vivo tumor formation and angiogenesis assays, the xenograft model of PCa was established according to our previous descriptions (Additional file 2: S1-section 4) [16–18]. Five weeks later for miR-30d and miR-NC PCa cells while seven weeks later for sh-30d and sh-NC, tumors were removed, fixed in formalin, and embedded in paraffin. Expression patterns of vascular endothelial growth factor A (VEGFA) and CD31 proteins in different groups were respectively detected by Western blot analysis and immunohistochemistry. The microvessel density (MVD) in tumor tissues was evaluated based on the immunostaining for CD31.

### Gene expression profiling

To identify the differentially expressed genes (DEGs) in LNCaP and DU145 cells transfected with miR-30d/miR-NC vectors, total RNA were amplified, labeled and purified by using GeneChip 3’IVT Express Kit (Cat#901229, Affymetrix, Santa Clara, CA, US) followed the manufacturer’s instructions to obtain biotin labeled cRNA. Array hybridization and wash was performed using GeneChip® Hybridization, Wash and Stain Kit (Cat#900720, Affymetrix, Santa Clara, CA, US) in Hybridization Oven 645 (Cat#00-0331-220 V, Affymetrix, Santa Clara, CA, US) and Fluidics Station 450 (Cat#00-0079, Affymetrix, Santa Clara, CA, US) followed the manufacturer’s instructions. Slides were scanned by GeneChip® Scanner 3000 (Cat#00-00212, Affymetrix, Santa Clara, CA, US) and Command Console Software 3.1 (Affymetrix, Santa Clara, CA, US) with default settings. Raw data were normalized by MAS 5.0 algorithm, Gene Spring Software 11.0 (Agilent technologies, Santa Clara, CA, US). The microarray data (ID: GSE85884) were deposited in Gene Expression Omnibus (GEO, http://www.ncbi.nlm.nih.gov/geo/). Then, significant DEGs were identified between the test and control groups using the criteria of P value <0.05 and |log2 fold change (FC)| > 0.5 with the R package (version 1.0.2, R Core Team, Vienna, Austria).

### Prediction of target genes of miR-30d

Three online programs Target-Scan (release 6.2) [19], miRWalk (Last Update: March 29, 2011) [20], and miRanda (August 2010 Release, Last Update: November 01, 2010) [21] were used to predict potential target genes for miR-30d.

### Luciferase reporter assay

To verify the binding site of miR-30d and its candidate target gene MYPT1, the luciferase reporter assay was performed according to our previous descriptions (Additional file 2: File S1-section 5) [16–18].

The article "MicroRNA-30d promotes angiogenesis and tumor growth via MYPT1/c-JUN/VEGFA pathway and predicts aggressive outcome in prostate cancer" was retracted in 2023. Reasons: duplicated images; unreliable results or conclusions.

### qRT-PCR

Expression levels of miR-30d, CALD1, TNPO1, ATP2B1, SEPT7, MYPT1, ZNF148, CEP350, KIF5B, STAG2 and GALNT1 mRNA in PCa cell lines and clinical PCa tissues were detected by qRT-PCR analysis according to our previous descriptions [16–18]. The sequences of all the primers are provided in Additional file 3: Table S1.

### Western blot analysis

Expression levels of MYPT1, total-c-JUN, p-c-JUN (ser63), p-c-JUN (ser73) and VEGFA proteins in PCa cell lines and clinical PCa tissues were detected by Western blot analysis according to the protocol of our previous studies [16–18]. The antibodies are provided in Additional file 3: Table S2.

### Immunohistochemistry

Cellular distribution and expression level of MYPT1 protein in clinical PCa tissues, and those of CD31 protein in subcutaneous tumor xenografts of nude mice were examined by immunohistochemistry according to our previous description [16–18]. The antibodies used in this study were shown in Additional file 3: Table S2.

### Statistical analyses

All statistical analyses were performed by SPSS software for Windows (version 17.0, SPSS Inc, IL, USA). Data of continuous variables were expressed as mean ± S.D. Data obtained from qRT-PCR and Western blot were conducted using Wilcoxon signed-rank test. Associations of miR-30d/MYPT1 expression with various clinicopathological parameters were evaluated by Fisher’s exact test for any 2 × 2 tables and Pearson *χ* ^2^ test for non-2 × 2 tables. Survival analysis was performed by Kaplan-Meier method and Cox regression model. Correlation between miR-30d and MYPT1 expression in clinical PCa tissue samples was assessed by the Spearman correlation analysis. For functional analyses in vitro and in vivo, the differences between groups were analyzed using a Student *t* test when comparing only two groups or one-way analysis of variance when comparing more than two groups. Differences were considered statistically significant when the *P* value was less than 0.05.

## Results

### miR-30d over-expression associates with advanced progression and unfavorable prognosis in human PCa

Compared to adjacent non-cancerous prostate tissues and normal human prostate epithelial cells, the expression levels of miR-30d were respectively increased in PCa tissues and two PCa cell lines (all *P* < 0.05, Additional file 1: Figure S2).

Associations of miR-30d expression with various clinicopathological parameters and patients’ prognosis of PCa were evaluated based on publicly available Taylor and TCGA datasets. PCa patients with high pre-operative PSA (for Taylor: *P* = 0.003) and Gleason score (for Taylor and TCGA: *P* = 0.010 and 0.001, respectively), advanced clinical (for Taylor: *P* = 0.007) and pathological stages (for Taylor: *P* = 0.004), and positive metastasis (for Taylor: *P* = 0.001) and biochemical recurrence (BCR, for Taylor and TCGA: *P* = 0.002 and 0.037, respectively) more frequently had higher expression level of miR-30d than those in the corresponding control groups (Additional file 3: Table S3). In survival analysis based on the Taylor dataset, all 113 PCa patients were divided into two groups (miR-30d-low, *n* = 57; miR-30d-high, *n* = 56) by setting cut-off value at the median miR-30d expression level. Then, pairwise comparisons showed significant differences in the BCR-free survival (*P* = 0.001, Fig. 1a) and overall survival (*P* = 0.041, Fig. 1a) between patients with high and low miR-30d expressions. Further univariate analysis using a COX regression model revealed that miR-30d expression was significantly correlated with BCR-free survival of PCa patients (Additional file 3: Table S4). Although the PCa patients in high miR-30d expression group had a trend of short BCR-free survival based on TCGA dataset, there was no statistical significance, due to a relative small BCR positive cohort in this dataset (Fig. 1a).

The article "MicroRNA-30d promotes angiogenesis and tumor growth via MYPT1/c-JUN/VEGFA pathway and predicts aggressive outcome in prostate cancer" was retracted in 2023. Reasons: duplicated images; unreliable results or conclusions.

**Fig. 1:** Prognostic value of miR-30d expression in PCa patients and its functions on tumor growth and angiogenesis in vivo using LNCaP cell induced tumor xenografts. **a** Kaplan-Meier analyses of biochemical recurrence (BCR)-free survival and overall survival of PCa patients based on miR-30d expression in Taylor and TCGA datasets. **b** LNCaP cells stably expressing miR-30d formed significantly larger tumor nodules and remarkably speeded up tumor xenografts growth compared with the controls. Conversely, PCa cells that permanently suppressed miR-30d expression led to the smaller tumor nodules and the slower tumor growth compared with the control. **c** Immunohistochemical analysis using pan-endothelial marker CD31 antibody. **d** VEGFA protein expression in different groups detected by Western blot analysis. Data were presented as Mean ± SD. *P < 0.05. **P < 0.01

### miR-30d promotes tumor growth and angiogenesis in vivo

To further determine the roles of miR-30d in tumor growth and angiogenesis in vivo, LNCaP and DU145 PCa cell lines stably expressing miR-30d or control vector were subcutaneously implanted into nude mice. LNCaP (Fig. 1b) and DU145 (Additional file 1: Figure S3A and B) cells stably expressing miR-30d formed significantly larger tumor nodules and remarkably speeded up tumor xenografts growth compared with the controls. Conversely, PCa cells that permanently suppressed miR-30d expression led to the smaller tumor nodules and the slower tumor growth compared with the controls (for LNCap: Fig. 1b; for DU145: Additional file 1: Figure S3 A and B).

The article "MicroRNA-30d promotes angiogenesis and tumor growth via MYPT1/c-JUN/VEGFA pathway and predicts aggressive outcome in prostate cancer" was retracted in 2023. Reasons: duplicated images; unreliable results or conclusions.

Moreover, immunohistochemical analysis using pan-endothelial marker CD31 antibody were employed to evaluate the angiogenesis of the tumor xenografts. As a result, the immunostaining of CD31 protein in the tumor xenografts established by LNCaP (Fig. 1c) or DU145 (Additional file 1: Figure S3C) cells stably expressing miR-30d were remarkably stronger than that in the control group. Contrarily, the tumor xenografts established by sh-30d-transfected LNCaP (Fig. 1c) or DU145 (Additional file 1: Figure S3C) cells presented markedly weaker CD31 immunostaining than the control xenografts. Consistently, the microvessel density (MVD) levels in tumor tissues of the subcutaneous models bearing miR-30d- and sh-miR-30d-transfected PCa cells were significantly higher and lower than those of the respective controls (both P < 0.05, Fig. 1c and Additional file 1: Figure S3C), which were in line with the changes into VEGFA protein expression in different groups (both *P* < 0.05, Fig. 1d and Additional file 1: Figure S3D).

### miR-30d enhances the promoting effects of PCa cells on in vitro proliferation, migration, invasion, and increases the abilities of PCa cells to recruit endothelial cells

QRT-PCR analysis confirmed that the expression levels of miR-30d in LNCaP cells transfected with a lentiviral vector expressing miR-30d and sh-30d were respectively higher and lower than those with miR-NC and sh-NC vectors (Additional file 1: Figure S4A), which were similar with the findings of DU145 cells (Additional file 1: Figure S5A).

CCK-8 assays indicated that the cellular proliferation of miR-30d-introduced LNCaP (Additional file 1: Figure S4B) and DU145 cells (Additional file 1: Figure S5B) were both significantly higher than those of control vectors-transfected cells (all *P* < 0.05), while the knockdown of miR-30d expression dramatically decreased the cell viability (all *P* < 0.05, Additional file 1: Figure S4B and S5B).

Transwell assays clearly revealed that enforced expression of miR-30d significantly enhanced the invasive activities of both LNCaP (Additional file 1: Figure S4C) and DU145 (Additional file 1: Figure S5C) cells, which were reduced by loss of miR-30d distinctly (Additional file 1: Figure S4C and S5C, all *P* < 0.05).

Wound-healing assays demonstrated that miR-30d upregulation markedly strengthened the migratory abilities of both LNCaP (Additional file 1: Figure S4D) and DU145 (Additional file 1: Figure S5D) cells, which were also suppressed by the transfection of sh-miR-30d vector (Additional file 1: Figures S4E and S5E, all *P* < 0.05).

The article "MicroRNA-30d promotes angiogenesis and tumor growth via MYPT1/c-JUN/VEGFA pathway and predicts aggressive outcome in prostate cancer" was retracted in 2023. Reasons: duplicated images; unreliable results or conclusions.

To assess the influence of miR-30d in the abilities of PCa cells to recruit endothelial cells, the condition medium of the PCa cells was collected and the transwell, wound healing and tube formation assays were performed. As a result, the culture medium of miR-30-transfected LNCaP (Fig. 2) and DU145 (Additional file 1: Figure S6) cells significantly enhanced the invasive and migrated abilities of HUVECs, and also promoted their capillary tube formation. In contrast, the medium of sh-miR-30d-transfected LNCaP (Fig. 2) and DU145 (Additional file 1: Figure S6) cells induced obvious decreases in the abilities of HUVEC invasion, migration and capillary tube formation.

**Fig. 2:** miR-30d enhances the capillary tube formation of endothelial cells. **a** Transwell assays of the invasive abilities of HUVECs with the culture medium of miR-30 or sh-miR-30d-transfected LNCaP cells; **b** Wound-healing assays of the migrated abilities of HUVECs with the culture medium of miR-30 or sh-miR-30d-transfected LNCaP cells; **c** Capillary tube formation assays of HUVECs with the culture medium of miR-30 or sh-miR-30d-transfected LNCaP cells. Data were presented as Mean ± SD. *P < 0.05. **P < 0.01

### MYPT1 is a direct target of miR-30d

Gene expression profiles of miR-30d- and miR-NC-transfected LNCaP and DU145 cells were respectively detected and normalized. With the thresholds of *P* value <0.05 and |log2 FC| >0.5, a total of 146 DEGs were commonly identified in both LNCaP and DU145 cells, including three up-regulated DEGs and 143 down-regulated DEGs (Additional file 3: Table S5).

Then, three miRNA target predicting programs (Target-Scan, miRWalk, and miRanda) were used to identify the putative targets of miR-30d, and found that there were 36 putative targets of miR-30d which were also downregulated in both miR-30d-transfected LNCaP and DU145 cells according to the gene microarray analysis (Additional file 3: Table S6 and Fig. 3a).

**Fig. 3:** MYPT1 functions as a critical downstream mediator of miR-30d's oncogenic effects in PCa progression. **a** Intersections among gene microarray identification and bioinformatics miRNA target prediction algorithm. **b** QRT-PCR analysis was performed detect the endogenous expression levels of SEPT7, MYPT1, ZNF148, CEP350, STAG2 and GALNT1 in miR-30d-transfected LNCaP cells. **c** Luciferase activity assays was performed to confirm the direct binding efficiency of miR-30d and its putative target MYPT1; **d** Western blot analysis was performed to detect the expression levels of MYPT1 protein in LNCaP cells transfected by lentivectors and in the tumor xenografts established by these LNCaP cells; **e** ~ **h** MYPT1 simulation antagonized the increasing effects on the abilities of migration, invasion, and capillary tube formation of HUVECs induced by miR-30d up-regulation in LNCaP cells. Data were presented as Mean ± SD. *P < 0.05. **P < 0.01

After the pathway enrichment analysis based on KEGG database, we found that the above 36 putative targets of miR-30d were significantly associated with several tumor-related pathways, such as RhoA signaling, DNA methylation and transcriptional repression signaling, Signaling by Rho family GTPases and PI3K/AKT signaling (Additional file 3: Table S7 and Additional file 1: Figure S7), which all have broad effects on cell behavior.

The article "MicroRNA-30d promotes angiogenesis and tumor growth via MYPT1/c-JUN/VEGFA pathway and predicts aggressive outcome in prostate cancer" was retracted in 2023. Reasons: duplicated images; unreliable results or conclusions.

In addition, qRT-PCR analysis was performed and the results showed that the endogenous expression levels of SEPT7, MYPT1, ZNF148, CEP350, STAG2 and GALNT1 in miR-30d-transfected LNCaP (Fig. 3b) and DU145 (Additional file 1: Figure S8A) cells were all significantly reduced at mRNA levels (*P* < 0.05). Among them, only MYPT1 is a major component in RhoA signaling pathway, which was one of the significantly enriched pathways involved by miR-30d-induced differentially-expressed proteins. Accumulating studies have reported that RhoA signaling pathway plays an important role in tumorigenesis and cancer metastasis [22]. Thus, MYPT1 would be selected as a candidate target for further analyses.

To confirm MYPT1 being targeted by miR-30d, the luciferase reporter containing the complimentary seed sequence of miR-30d at the 3’-UTR regions of MYPT1 mRNA was constructed. Luciferase activity assays showed that the expression of the MYPT1 reporter was significantly reduced by co-transfection with has-miR-30d mimics. In contrast, the expression of the MYPT1 reporter containing the mutated sequence of the same fragment was not affected by co-transfection with hsa-miR-30d mimics (Fig. 3c). The results indicated that the fragment at the 3'-UTR of MYPT1 mRNA was the complementary site for the miR-30d seed region, suggesting that MYPT1 may be a direct target of miR-30d.

### MYPT1 functions as a critical downstream mediator of miR-30d's oncogenic effects in PCa progression

We performed western blot to detect the expression levels of MYPT1 protein in LNCaP and DU145 cells transfected by lentivectors and in the tumor xenografts established by these PCa cells. MYPT1 protein levels were remarkably down-regulated in LNCaP (Fig. 3d) or DU145 (Additional file 1: Figure S8B) cells stably overexpressing miR-30d. The similar findings were observed in the corresponding tumor xenografts established by cell lines overexpressing miR-30d (Fig. 3d and Additional file 1: Figure S8B). In contrast, the expression levels of MYPT1 protein in sh-miR-30d-transfected cell lines and the corresponding tumor xenografts were all significantly up-regulated (Fig. 3d and Additional file 1: Figure S8B). Overall, miR-30d negatively regulated MYPT1 expression in vitro and in vivo.

The article "MicroRNA-30d promotes angiogenesis and tumor growth via MYPT1/c-JUN/VEGFA pathway and predicts aggressive outcome in prostate cancer" was retracted in 2023. Reasons: duplicated images; unreliable results or conclusions.

To clarify whether the roles of miR-30d in PCa were mediated through suppressing MYPT1 expression, pCDNA3.1(+)-Vectors expressing MYPT1 were conducted. As shown in the Fig. 3e ~ h, Additional file 1: Figure S8C ~ D and Figure S9, MYPT1 simulation antagonized the increasing effects on the abilities of migration, invasion, and capillary tube formation of HUVECs induced by miR-30d up-regulation in PCa cells.

### miR-30d/MYPT1 combination is a more efficient prognostic factor for BCR-free survival of PCa patients than miR-30d or MYPT1 alone

On the basis of our clinical cohort of PCa sample tissues, the Taylor and TCGA datasets, the Spearman Correlation analysis clearly presented a negative correlation between MYPT1 mRNA and miR-30d expression in PCa tissues (for our clinical cohort: Fig. 4a, for Taylor and TCGA datasets: Additional file 1: Figure S10).

**Fig. 4:** miR-30d/MYPT1 combination is a more efficient prognostic factor for BCR-free survival of PCa patients than miR-30d or MYPT1 alone. **a** Correlation between MYPT1 mRNA and miR-30d expression in PCa tissues was evaluated by Spearman Correlation analysis; **b** Immunohistochemical staining images of MYPT1 protein in adjacent non-cancerous prostate tissues and PCa tissues with different Gleason scores; **c** The immunoreactive scores (IRS) of MYPT1 protein in PCa clinical samples and adjacent benign tissues; **d** and **e** Kaplan-Meier analysis on the associations between MYPT1 expression and BCR-free survival, overall survival and metastasis-free survival; **f** Kaplan-Meier analysis on the associations between miR-30d/MYPT1 combination and BCR-free survival and overall survival of PCa patients using the Taylor dataset

To investigate whether MYPT1 expression could be linked to the clinicopathological features of human PCa, the immunohistochemical staining was employed to detect the expression pattern and subcellular localization of MYPT1 expression in 225 PCa and 25 adjacent non-cancerous prostate tissues. As shown in Fig. 4b, the antibody that specifically recognizes MYPT1 stained the cytoplasm and cellular membrane of PCa cells, and gave evenly distributed staining pattern with various intensities. The immunoreactive scores (IRS) of MYPT1 protein in PCa clinical samples was significantly lower than that in adjacent benign tissues (*P* < 0.001, Fig. 4c). Interestingly, MYPT1 protein expression in PCa tissues displayed a decreasing trend depend on the increasing Gleason scores (*P* < 0.05, Fig. 4c) and the presence of BCR (*P* < 0.05, Fig. 4c).

The article "MicroRNA-30d promotes angiogenesis and tumor growth via MYPT1/c-JUN/VEGFA pathway and predicts aggressive outcome in prostate cancer" was retracted in 2023. Reasons: duplicated images; unreliable results or conclusions.

Then, the data shown in Additional file 3: Table S8 revealed that low IRS of MYPT1 protein was significantly associated with high Gleason score (*P* = 0.002), positive metastasis (*P* = 0.018) and BCR (*P* < 0.001) and shorter overall survival (*P* = 0.005) of PCa patients. Kaplan-Meier analysis showed that there were significant differences in the BCR-free survival (P < 0.001, Fig. 4d), overall survival (*P* = 0.005, Fig. 4d) and metastasis-free survival (*P* = 0.005, Fig. 4d), between patients with high and low MYPT1 expression. Notably, regarding to the PCa patients with Gleason score = 7, low MYPT1 expression was significantly associated with short BCR-free survival (*P* = 0.037, Fig. 4*e*). In addition, the prognostic potential of miR-30d/MYPT1 combination in BCR-free survival of PCa patients was also confirmed using the Taylor dataset (*P* = 0.003, Fig. 4f). Further Cox proportional hazards multivariate model revealed that the prediction efficiency of miR-30d/MYPT1 combination to BCR of PCa patients was stronger than the two markers’ alone (For prognostic implication of MYPT1 based on its immunostainings using human PCa tissue microarrays: Table 1; For prognostic implications of miR-30d and/or MYPT1 based on the Taylor dataset: Additional file 3: Table S9, P value of miR-30d/MYPT1 combination for BCR-free survival vs. P values of miR-30d or MYPT1: 0.026 vs. 0.027 or 0.624).

**Table 1:** Prognostic value of MYPT1 expression for the biochemical recurrence-free, metastasis-free and overall survival in univariate and multivariate analysis using Cox Regression models

	Univariate			Multivariate		
	HR	95% Cl	P	HR	95% Cl	P
Time to BCR						
MYPT1 (high vs low)	0.371	0.232–0.593	<0.001	0.468	0.282–0.775	0.003
Tumor stage (T2 vs T3)	1.879	1.207–2.925	0.005	1.123	0.668–1.888	0.661
Surgical margin (+ vs -)	1.805	1.185–2.749	0.006	1.124	0.673–1.876	0.655
Gleason score (<8 vs ≥8)	4.541	2.832–7.280	<0.001	3.482	2.010–6.033	<0.001
Pre-operative PSA (<4 vs ≥4)	1.792	1.090–2.947	0.022	1.941	0.877–4.300	0.102
Age (<66 vs ≥66)	1.502	0.973–2.320	0.067	1.361	0.848–2.183	0.201
Time to Metastasis						
MYPT1 (high vs low)	0.376	0.137–1.035	0.058	0.420	0.148–1.191	0.103
Tumor stage (T2 vs T3)	1.574	0.628–3.946	0.333	1.179	0.401–3.464	0.764
Surgical margin (+ vs -)	0.963	0.394–2.356	0.934	0.608	0.208–1.781	0.364
Gleason score (<8 vs ≥8)	4.765	1.945–11.672	0.001	3.563	1.258–10.094	0.017
Pre-operative PSA (<4 vs ≥4)	1.780	0.676–4.684	0.243	0.577	0.202–1.649	0.305
Age (<66 vs ≥66)	0.940	0.361–2.448	0.900	0.744	0.265–2.091	0.575
Time to Death						
MYPT1 (high vs low)	0.375	0.183–0.768	0.007	0.334	0.150–0.742	0.007
Tumor stage (T2 vs T3)	1.626	0.852–3.103	0.140	1.305	0.604–2.823	0.498
Surgical margin (+ vs -)	1.178	0.636–2.183	0.603	0.534	0.250–1.142	0.106
Gleason score (<8 vs ≥8)	4.033	2.111–7.705	<0.001	2.941	1.335–6.477	0.007
Pre-operative PSA (<4 vs ≥4)	1.275	0.600–2.713	0.527	1.045	0.388–2.814	0.931
Age (<66 vs ≥66)	1.818	0.980–3.369	0.058	1.876	0.952–3.695	0.069

*HR* Hazard ratio, *CI* confidence interval; Surgical margin status, between positive and negative

The article "MicroRNA-30d promotes angiogenesis and tumor growth via MYPT1/c-JUN/VEGFA pathway and predicts aggressive outcome in prostate cancer" was retracted in 2023. Reasons: duplicated images; unreliable results or conclusions.

### miR-30d promotes angiogenesis via MYPT1/c-JUN/VEGFA pathway in PCa

The above data indicated an important role of miR-30d/MYPT1 axis in tumor angiogenesis of PCa in vitro and in vivo, which prompted us to investigate the underlying molecular mechanisms. As a potent endothelial mitogen, VEGFA has been demonstrated to be crucial for cancer growth and neovascularization [23]. Our data mentioned above showed that miR-30d up-regulation could increase the expression level of VEGFA protein in PCa cell lines and in tumor tissues of the subcutaneous models. The VEGFA promoter region includes several candidate binding sites for the transcription factors, such as hypoxia inducible factor-1α (HIF-1α), activator protein-1 (AP-1, c-JUN), AP-2 and Specificity protein-1 (SP-1) [24]. Thus, we firstly transfected si-HIF-1α, si-c-JUN, si-AP-2 and si-SP-1 into LNCap and DU145 cells, and found that the loss of HIF-1α, AP-2 and c-JUN transcription activities significantly inhibited the expression level of VEGFA protein (Fig.5a and Additional file 1: Figure S11A). Since MYPT1 functions as targeting and regulatory subunits to confer substrate specificity and subcellular localization on the catalytic subunit of type 1d protein serine/threonine phosphatase [25], we hypothesized that the pro-angiogenic role of miR-30d might be related to the effect of MYPT1 on the activation of c-JUN and the expression of VEGFA. To verify this hypothesis, western blot analysis was performed to detect the expression levels of total-c-JUN, p-c-JUN (ser63), p-c-JUN (ser73) and VEGFA proteins in LNCap and DU145 cells transfected with miR-30d expressing or si-MYPT1 vectors. As shown in Fig.5b ~ f and Additional file 1: Figure S11B ~ F, both the enforced expression of miR-30d and the knockdown of MYPT1 significantly activated c-JUN and increased the expression of VEGFA protein, implying that c-JUN and VEGFA might function as the downstream effectors of miR-30d-MYPT1 axis in human PCa cells and be implicated in tumor angiogenesis during PCa progression.

**Fig. 5:** miR-30d promotes angiogenesis via MYPT1/c-JUN/VEGFA pathway in PCa: **a** Expression levels of VEGFA protein in LNCaP cells transfected si-HIF-1α, si-c-JUN, si-AP-2 and si-SP-1 detected by western blot analysis; **b** ~ **f** Expression levels of MYPT1, VEGFA, total-c-JUN, p-c-JUN (ser63), p-c-JUN (ser73) proteins in LNCaP cells transfected with miR-30d expressing or sh-MYPT1 vectors detected by western blot analysis. Data were presented as Mean ± SD. *P < 0.05. **P < 0.01

The article "MicroRNA-30d promotes angiogenesis and tumor growth via MYPT1/c-JUN/VEGFA pathway and predicts aggressive outcome in prostate cancer" was retracted in 2023. Reasons: duplicated images; unreliable results or conclusions.

## Discussion

Growing evidence show that active angiogenesis, a critical step in cancer development and progression, is responsible for the rapid recurrence and poor prognosis of patients with PCa [26]. Dysfunction of miRNAs in malignant cells has been revealed to play important roles in tumor angiogenesis [27, 28]. In the current study, we identified the pro-angiogenic function of miR-30d in PCa for the first time using in vitro and in vivo assays. The elevated level of miR-30d expression was positively associated with aggressive progression and short BCR-survival of patients with PCa. Through up- and down-regulating miR-30d in PCa cells, we confirmed that miR-30d could efficiently enhance the abilities of in vitro proliferation, migration, invasion and capillary tube formation of HUVECs, as well as promote in vivo tumor growth and angiogenesis in nude mice models bearing human PCa. We also found that the pro-angiogenic effect of miR-30d might be due to its regulation on the direct target gene MYPT1, subsequently leading to the activation of c-JUN and the increased expression of VEGFA protein, a critical pro-angiogenic factor secreted by cancer cells.

The miR-30 family of miRNAs is involved in regulation of various physiological processes in normal and malignant tissues, such as epithelial-mesenchymal transition (EMT), which is a developmental program characterized by loss of cell adhesion and increased cell mobility, and is critical for embryogenesis and organ development [29]. Dysregulation of the miR-30 family members are found implicated in tumor development and progression; however, inconsistency exists about their function in various cancer types. For example, they have been identified as oncomiRNAs melanoma (miR-30b/d) [10], renal cancer (miR-30c) [30], hepatocellular carcinoma (miR-30d) [31], and glioma (miR-30e) [32]; In contrast, they function as tumor suppressors in breast cancer (miR-30a) [33], non-small cell lung cancer (miR-30b/miR-30c) [34], renal carcinoma (miR-30d) [35], and gastrointestinal cancer (miR-30c) [36]. As a member of this family, miR-30d has been identified as a novel cancer-related biomarker and a potential therapeutic target in multiple malignancies. It functions either as an oncomiR or a tumor suppressor depend on cancer types through regulating different target genes. The decreased expression of miR-30d was observed in chronic lymphocytic leukemia [37], thyroid cancer [38], renal carcinoma [35] and cervical cancer [39], and was associated with highly malignant phenotypes of these cancer cells; Conversely, the upregulation of miR-30d in hepatocellular carcinoma [31], medulloblastoma [40] and breast cancer [41] could promote the advanced progression of patients with these malignancies. Accumulating studies have identified a variety of target genes for miR-30d in different cancer cells. For example, miR-30d inhibited renal carcinoma cell proliferation via the regulation of cyclin E2 expression post-transcriptionally [35]; miR-30d enhanced the invasion and metastasis abilities of hepatocellular carcinoma cells by targeting Galphai2 [31]; Ectopic expression of miR-30d inhibited proliferation and colony formation of anaplastic thyroid carcinoma cells by inducing G2/M-phase cell-cycle arrest via regulating the Polycomb Protein EZH2 [42]. Due to these disparities in different cancer types, it is necessary to clarify the precise molecular mechanism underlying the involvement of miR-30d in various human cancers.

The article "MicroRNA-30d promotes angiogenesis and tumor growth via MYPT1/c-JUN/VEGFA pathway and predicts aggressive outcome in prostate cancer" was retracted in 2023. Reasons: duplicated images; unreliable results or conclusions.

Even though aberrant expression of miR-30d has been reported in PCa, its associations with cancer progression remain contradictory [11–15]. In the current study, we identified the upregulation of miR-30d as a characteristic molecular change in both PCa cell lines and clinical tissue samples, in line with the findings of Kobayashi group [11]. Then, we also confirmed the significant associations of miR-30d upregulation with aggressive clinicopathological characteristics, shorter BCR-free and overall survivals of PCa patients, which prompted us to determine the roles of miR-30d in malignant phenotypes of PCa in vitro systems and in vivo models. Our data showed the oncogenic role of miR-30d through PCa cells viability, migration, invasion and tube formation assays in vitro, along with tumor xenografts growth and angiogenesis in vivo according to both gain-of-function and loss-of-function experiments. We also found that the pro-angiogenic effects of miR-30d in PCa might be due to the upregulation of VEGFA. However, VEGFA was not a direct target gene of miR-30d according to our miRNA target gene identification. To elucidate the mechanisms underlying the regulatory effect of miR-30d on VEGFA expression in PCa cells, we combined gene expression profile, three miRNA target prediction algorithms, luciferase report assay, the correlation analysis in both PCa tissues and cell lines, with both in vitro and in vivo functional analyses, to confirm that miR-30d may exert its oncogenic role at least in part by suppressing MYPT1, which is involved into the Rho/Rho-kinase pathway [43]. The abnormal of this pathway may be associated with various pathological states, such as vascular spasm [44]. There was an inverse correlation between miR-30d and MYPT1 mRNA levels in PCa tissues, which was further confirmed by evaluating the effects of up- and down-regulating miR-30d on MYPT1 expression in PCa cells. In addition, MYPT1 stimulation could antagonize the effects of miR-30d, implying that MYPT1 may serve as a downstream mediator of miR-30d function in PCa. It has been reported that ROK phosphorylation of threonine 696 on MYPT1 may inhibit myosin phosphatase catalytic activity, which can modulate the motility of cancer and endothelial cells, and neoangiogenesis [45]. Here, our solid data of both LNCap and DU145 cells transfected with miR-30d expressing or si-MYPT1 vectors indicated that miR-30d upregulation and MYPT1 downregulation significantly promoted the activation of c-JUN which can bind to the VEGFA promoter and regulated VEGFA transcription directly. These provide further evidence to support that miR-30d may increase VEGFA expression by active MYPT1-cJUN pathway (Fig. 6).

The article "MicroRNA-30d promotes angiogenesis and tumor growth via MYPT1/c-JUN/VEGFA pathway and predicts aggressive outcome in prostate cancer" was retracted in 2023. Reasons: duplicated images; unreliable results or conclusions.

**Fig. 6:** Schematic diagram of the miR-30d- MYPT1-cJUN pathway

Another important finding of this study was that miR-30d and its direct target gene MYPT1, alone or in combination, were novel independent prognostic markers for BCR-free survival of patients with PCa. Especially, the Cox proportional hazards multivariate model based on the Taylor dataset revealed that the prediction efficiency of miR-30d/MYPT1 combination to BCR of PCa patients was stronger than the two markers’ alone. However, we found that the association between miR-30d expression and patients' BCR-free survival didn't have statistical significance based on the TCGA dataset, the reason for which might be a relative small BCR positive cohort in this dataset.

## Conclusions

Our data offer the promising evidence that miR-30d may function as an oncogene in human PCa by promoting tumor angiogenesis via regulating MYPT1/c-JUN/VEGFA pathway signaling. Our results supporting miR-30d and/or MYPT1 as promising prognostic markers which have potential implications for allowing clinicians to screen patients with intensive diseases. Considering anti-angiogenesis therapy is an important strategy of cancer treatment, miR-30d might be a novel therapeutic target for PCa.

## Additional files

Additional file 1: Figure S1. A schematic diagram of the systematic strategies for uncovering the involvement of miR-30d in human prostate cancer (PCa). **Figure S2.** miR-30d expression in human PCa cell lines (A) and clinical PCa tissues (B). Data were presented as Mean ± SD. ***P*<0.01. **Figure S3.** miR-30d promotes tumor growth and angiogenesis in vivo using DU145 induced tumor xenografts. **Figure S4.** miR-30d enhances proliferation, invasion and migration of LNCaP cells. **Figure S5.** miR-30d enhances proliferation, invasion and migration of DU145 cells. **Figure S6.** miR-30d enhances the capillary tube formation of endothelial cells. **Figure S7.** Functional enrichment analysis of putative targets of miR-30d. **Figure S8.** MYPT1 functions as a critical downstream mediator of miR-30d's oncogenic effects in PCa progression. **Figure S9.** The re-expression of MYPT1 could rescue the promoting effects of miR-30d on tumor angiogenesis in LNCaP and DU145 cells. **Figure S10.** Correlation between miR-30d and MYPT1 expression in prostate cancer (PCa) tissues based on the Taylor (A) and TCGA datasets (B). **Figure S11.** miR-30d promotes angiogenesis via MYPT1/c-JUN/VEGFA pathway in PCa. (DOCX 7972 kb)
Additional file 2:
**File S1.** for the manuscript titled as “MicroRNA-30d promotes angiogenesis and tumor growth via MYPT1/c-JUN/VEGFA pathway and predicts aggressive outcome in prostate cancer”. (DOC 38 kb)
Additional file 3: Table S1. The sequences of all the primers. **Table S2.** The antibodies of all proteins. **Table S3.** Associations of miR-30d expression with various clinicopathological parameters of PCa patients based on Taylor and TCGA datasets. **Table S4.** Univariate and multivariate analyses on prognostic implications of various clinicopathological parameters of human PCa based on Taylor dataset. **Table S5.** One hundred and forty-six differentially expressed gene with more than 2 ratio both in LNCaP and DU145 cells from gene expression profile. **Table S6.** Thirty-six putative targets of miR-30d which were also downregulated in both miR-30d-transfected LNCaP and DU145 cells according to the gene microarray analysis. **Table S7.** The pathway enrichment analysis based on KEGG database. **Table S8.** Associations of MYPT1 protein expression with clinicopathological characteristics of PCa patients. **Table S9.** Cox proportional hazards multivariate model for evaluating the prognostic values of various factors in human prostate cancer based on Taylor dataset. **Table S10.** Associations between MYPT1 expression in PCa tissues and Gleason score. **Table S11.** Associations between miR-30d expression in PCa tissues and Gleason score based on Taylor and TCGA datasets. (DOCX 58 kb)

The article "MicroRNA-30d promotes angiogenesis and tumor growth via MYPT1/c-JUN/VEGFA pathway and predicts aggressive outcome in prostate cancer" was retracted in 2023. Reasons: duplicated images; unreliable results or conclusions.

## Abbreviations

PCa: Prostate cancer
PSA: Prostate-specific antigen
miRNA: MicroRNAs
EMT: Epithelial-mesenchymal transition
